This article has been retracted.

# Effect of Endoscopic Retrograde Cholangiopancreatography Lithotomy Combined with Laparoscopic Cholecystectomy on Pain and Prognosis of Patients with Gallstones and Extrahepatic Bile Duct Stones

**DOI:** 10.1155/2022/9450159

**Published:** 2022-06-27

**Authors:** Hui Zhao, Jian Zhang

**Affiliations:** ^1^Department of Gastroenterology, Huzhou Central Hospital, Huzhou 313000, China; ^2^Department of Gastroenterology, Affiliated Central Hospital Huzhou University, Huzhou 313000, China; ^3^Department of Hepatobiliary Surgery, Huzhou Central Hospital, Huzhou 313000, China; ^4^Department of Hepatobiliary Surgery, Affiliated Central Hospital Huzhou University, Huzhou 313000, China

## Abstract

**Objective:**

The researchers aim to assess how endoscopic retrograde cholangiopancreatography lithotomy and laparoscopic cholecystectomy affected pain and prognosis in individuals with gallstones and extrahepatic bile duct stones.

**Methods:**

Researchers studied 100 persons with gallstones and extrahepatic bile duct stones from January 2016 to August 2021. They were split into two groups: control and observation. The control group underwent open cholecystectomy + choledocholithotomy + *T*-tube drainage. There were ERCP + lithotomy + Laparoscopic cholecystectomy procedures conducted on the observation group of patients (LC). The operation time, incision size, and bleeding volume; stone clearance rate and stone recurrence rate; visual analogue scale (VAS); Eating time, exhaust time, out of bed activity time, and postoperative hospital stay; the two groups' difficulties were contrasted and studied.

**Results:**

The observation group's operation duration was much longer than the control group's, and the incision size and bleeding volume were significantly reduced in the observation group. When it came to recurrence, there was a significant difference between the observation group (2.0%) and the control group (4.0%), even though stone clearance did not differ substantially (20.00%). The VAS scores 3 and 7 days after surgery were significantly different between the observation and control groups. The observation group's eating time, exhaustion, activity time, and postoperative hospital stay were much shorter than the control group's; complications occurred at a lower rate (20%) in the observation group than in the control group (34%).

**Conclusion:**

When gallstones and extrahepatic bile-duct stones are removed using laparoscopic lithotomy and laparoscopic cystoscopy (LC), the operation indices are improved and the risk of recurrence of stones is reduced and reducing the occurrence of complications, all of which improve patient outcomes and deserve to be considered a clinical reference.

## 1. Introduction

Gallstone is a common clinical gallbladder disease, mainly manifested as biliary colic, continuous distention pain, right upper abdominal pain, etc. [1]. Relevant studies have shown that about 10% ∼ 15% of patients with cholecystolithiasis are also complicated with extrahepatic bile duct stones, which requires timely treatment; otherwise, it is likely to lead to a liver abscess, cirrhosis, acute bile duct obstruction, and other serious complications, increasing the difficulty of clinical treatment [2]. Patients with cholecystolithiasis complicated with extrahepatic bile duct stones are generally treated with surgery. In addition, surgery is mainly to remove stones and relieve clinical symptoms of patients [3]. In the past, the laparotomy method was adopted, although the curative effect was remarkable. However, its surgical trauma is large, patients recover slowly, and upper *T* tube drainage may cause bile duct bleeding and bile loss [4]. As science and medical technology have progressed, minimally invasive therapies have become increasingly common. Meanwhile, endoscopic retrograde cholangiopancreatography (ERCP) + lithotomy is a commonly used treatment at present. First of all, ERCP can intuitively and completely display the angiographic images of the biliary tract, which is conducive to a surgical operation. Using ERCP + lithotomy can help avoid incisions of the common bile channel, reduce difficulties, and reduce consequences. For the treatment of gallstones, laparoscopic cholecystectomy (LC) is well acknowledged [5]. More research is needed, however, to determine whether or not the combined use of ERCP + lithotomy and LC is effective in treating cholecystic bile duct stones, which can worsen the condition. For this study's main objective, researchers will look at how ERCP + LITHOMOY combined with the LC procedure affects the pain and prognosis of cholecystolithiases and extrahepatic bile duct stones patients, in order to provide more information for the clinical treatment of cholecystolithiases and extrahepatic bile duct stones patients.

## 2. Methods and Data

### 2.1. Information in General

With a random number table, 100 individuals with both cholecystolithiasis and extrahepatic stone disease were selected for this investigation, which lasted from January 2016 to August 2021. The observation group had ERCP + stone extraction combined with LC, while the control group received cholecystectomy + choledocholithotomy + *T* tube drainage. This research was authorized by the hospital's ethics committee. For example, there was no significant difference in the number of bile duct stones or stone diameter between the two groups as shown in Table 1.

### 2.2. Criteria for Inclusion and Removal

Inclusion criteria [6]: ① all patients were diagnosed with cholecystolithiasis and extrahepatic bile duct calculi using computed tomography, B ultrasonography, magnetic resonance cholangiopancreatography (MRCP), and other procedures; (2) patients with healthy organs such as the heart, liver, and kidneys; ③ extrahepatic bile duct stone diameter <2 cm; ④ written permission was obtained from patients or their guardians.

Exclusion criteria [7]: ① patients who cannot have surgery due to medical reasons or physical incapacity are included in this study; ② patients with abnormal biliary anatomic structure; ③ patients with other bile duct and biliary tract diseases; ④ patients with duodenum, hepatobiliary, and gastric surgery history; ⑤ patients with severe abdominal adhesion; ⑥ patients who suffer from a disorder of coagulation; ⑦ patients that have cancerous growths on their bodies.

## 3. Methods

The control group received open cholecystectomy + choledocholithotomy + *T* tube drainage: the patients were first given general anesthesia and then supine on the operating table. The four-hole method was used for cholecystectomy. Surgeons were able to remove it from the xiphoid process, which was attached to the common bile duct's anterior wall, and the fibrous catheter was implanted from 10 millimeters below. The stone was removed with a stone basket and pulled out directly from the puncture sheath. After the completion of stone removal, a routine examination of the extrahepatic bile duct was performed to avoid residual stones, and then catheterization was conducted from ventrofora to the right abdominal wall. The common bile duct was left with a No. 22 or 20 T tube in place when the operation was completed. The long arm of *T* tube extracted from puncture hole beneath the right costal edge, also known as the xiphoid process.

The observation group received ERCP + lithotomy combined with LC: the patients were first given general anesthesia and then made to lie on the side of the operating table. The duodenoscope was inserted through the mouth and 30% meglumine was injected for retrograde cholangiography. The size, number, hardness, location, and anatomical structure of the calculi were observed, and the mastoid muscle was cut 10 ∼ 15 mm. The net basket lithotomy was performed under the endoscope by electric cutting and coagulation mixed current. First, the balloon or stone basket is inserted for stone removal. For stones with a diameter of >1 cm, a mechanical gravel basket can be used for stone removal. Then, according to the residual calculus, the decision is whether to indurate nasobiliary drainage. LC should be performed 2 to 5 days after the patient's condition becomes stable after surgery. If necessary, somatostatin or protease inhibitors are administered to address the patient's elevated amylase levels. The three-hole approach was used to dissect the gallbladder triangle, and the gallbladder duct should be treated first before cholecystectomy to avoid gallbladder stones from entering the common bile duct. The gallbladder was removed after it had been removed, that is, to confirm whether there is residual bile or bleeding in the abdominal cavity. If there is no abnormality, the abdominal cavity is washed with sterilized injection water, the surgical instruments is withdrawn , the incision is sutured, and the abdominal cavity is closed.

Two groups of patients were given routine anti-infection therapy, nutritional support, fluid replenishment, maintenance of acid-base, and electrolyte balance.

### 3.1. Observation Indicators

① The length of the procedure, the size of the incision, and the amount of blood loss were all compared between the two groups. ② Treatment effects were evaluated by comparing how often stones were removed and how often they returned across the two groups.③ Prior to surgery, three days following surgery and seven days following surgery, patients in both groups had their pain levels evaluated using the Visual Analogue Scale (VAS) [8]. A perfect 10 was awarded for each measurement. The worse the pain, the higher the score. ③ Postoperative recovery: in terms of feeding time, exhaustion time, ambulation time, and postoperative hospital stay, the two groups were compared; complications: postoperative pancreatitis, hyperamylasemia, abdominal infection, bleeding, biliary fistula, etc., were observed in the two groups.

### 3.2. Statistical Methods

For the statistical analysis, we used SPSS 18.0. The measurement data were expressed as mean ± standard deviation (±*S*) and tested by *T*. *P* < 0.05 indicated a statistically significant difference.

## 4. Results

### 4.1. Comparison of Surgical Indicators

This study showed statistically significant differences between the observation group and the control group with regard to operation time, incision size, and blood loss (Table 2).

### 4.2. Comparison of Therapeutic Effects

Neither group's stone clearance rate (*P* > 0.05) was significantly different from the control group's; however, the observation group's stone recurrence rate (Table 3) was significantly lower.

### 4.3. Pain Level Comparison

Prior to surgery, there was no statistically significant difference in VAS values. While both groups had decreased VAS ratings at 3 and 7 days after surgery, at three and seven days following surgery, the VAS ratings of patients in the observation group were lower than those of patients in the control group, according to Table 4 and Figure 1.

### 4.4. Comparison of Postoperative Recovery

Feeding time, fatigue time, ambulation time, and postoperative hospitalization duration were all statistically different between the observation and control groups (Table 5).

### 4.5. Comparison of Complications

Table 6 shows that the observation group had a statistically significant (*P* < 0.05) lower incidence of complications than the control group.

## 5. Discussion

Extrahepatic bile duct stones induce stomach pain in cholecystolithiasis accompanied by extrahepatic bile duct stones. Its prevalence is increasing as society ages, posing a severe threat to human health and quality of life. Although traditional open surgery has a definite curative effect, it is more traumatic, with a slower prognosis and more complications [9]. With the progress of science and technology, minimally invasive technology gradually entered into clinical treatment and began to replace the traditional operation. ERCP + lithotomy has little trauma, low operation difficulty, and fewer complications [10]. LC magnifies the lesion through laparoscopic technology, which is convenient for the operator to observe and operate. At the same time, it is less traumatic and patients can obtain a good prognosis [11]. Extrahepatic bile duct stones occur in people with cholecystolithiasis, and only a few studies have examined the effects of ERCP + lithotomy combined with LC on their discomfort and prognosis. These patients may be better served by ERCP + lithotomy and LC in the study's findings, according to the researchers. This is for a number of reasons: Hajibandeh et al. [12] found that after combining ERCP and LC therapy, Roux-EN-Y gastric bypass patients had a success rate of 95.9 percent when it came to remove stones. The observation group's stone clearance rates were much greater than the control group's, while the observation group's stone recurrence rates were significantly lower. At the same time, this study discovered that the observation group's incision size and blood loss were lower than the control group's and that the operation time was longer than the control group's. Combined with the above-given results, ERCP + lithotomy combined with LC can effectively treat gallstones and improve a number of surgical indicators. To begin, the typical surgical procedure necessitates the complete separation and dissection of the common bile duct, as well as the incision of the front wall of the common bile duct. After the common bile duct incision, choledochoscope is used to explore the stone through the incision, which increases the surgical trauma and leads to bleeding [13]. ERCP has a high diagnostic efficiency for biliary and pancreatic diseases. It can clearly display the lesions of the bile duct and itself, the location and shape of calculi, and observe the location, degree, and nature of the lesions, so as to effectively remove calculi, reduce residual and reduce the risk of recurrence [14]. Compared with traditional surgery, the application of ERCP + lithotomy avoids the incision of the common bile duct and reduces iatrogenic injury. Moreover, it is a minimally invasive operation with a small incision and less trauma. The observation group's operation time was longer than the control group's due to the complexity and difficulty of ERCP + lithotomy combined with LC [15, 16].

Patients with cholecystolithiasis and extrahepatic bile duct stones commonly have biliary colic, chronic distention pain, and right upper abdomen pain. Therefore, reducing the pain degree of patients is one of the important objectives of clinical treatment [17]. Laparoscopic-assisted ERPC can successfully reduce pain in gastric bypass patients, according to Mohammad et al. [18]. In this study, after treatment, the VAS ratings of both the observation and control groups were significantly lower than in the other groups. In patients with cholecystolithiasis and other bile-duct stones, ERCP + lithotomy combined with LC can greatly relieve discomfort, according to the results of Mohammad's study. Efficient stone removal is possible in individuals with extrahepatic bile-duct stones when ERCP + lithotomy is used in conjunction with the procedure. At the same time, it also effectively expands the application range of minimally invasive surgery in biliary surgery, without *T* tube drainage, which not only ensures the normal physiological function of the digestive tract and biliary integrity but also reduces the pain of patients. In addition, ERCP + lithotomy combined with LC, as a minimally invasive surgery, has little trauma, can effectively reduce unnecessary injuries, and avoid water, electrolyte, and physiological dysfunction caused by bile outflow, which is beneficial to relieve patients' pain [19, 20].

Reversible electroporation did not cause pancreatitis in individuals with locally advanced pancreatic cancer after ERCP, according to Bhutiani et al. [21]. Compared to the control group, the observation group's feeding times, fatigue periods, and out-of-bed activity times were all considerably shorter. The rate of complications in the experimental group was much lower than in the control group. It was found in the Bhutiani study that patients with extrahepatic bile duct stones who had ERCP + lithotomy and LC had improved prognoses. The reasons were analyzed: postoperative recovery of patients was closely related to intraoperative trauma and blood loss, etc. Compared with traditional surgical methods, related indicators of ERCP + lithotomy combined with LC were better. As a result, overall function recovery time is decreased, and postoperative hazards are reduced. At the same time, cholecystectomy + choledochotomy for stone removal is easy to be complicated with infection, biliary fistula, and bleeding, while ERCP + stone removal combined with LC does not require choledochotomy, so it can effectively reduce the occurrence of multiple complications [22, 23].

The sample size used for this study is tiny, which may cause the data in the result to diverge from the actual value to some extent. As a result, the sample size should be increased in order to conduct additional verification investigations. For these reasons and more, it is recommended that patients who have been diagnosed with cholecystolithiasis or extrahepatic bile duct stones undergo an operation that includes ERCP + lithotomy in addition to liver cystoscopy and liver cystoscopy. These procedures have been shown to reduce the risk of recurrence, decrease pain, and speed up recovery time following surgery. [24, 25].

## Figures and Tables

**Figure 1:** Comparison of pain degree. *Note.* Before the operation, ^*∗*^*P* < 0.05; Compared to the control group, ^#^*P* < 0.05.

**Table 1:** A comparison of two generic data groups.

Indicators		Control group (*n* = 50)	Observation group (*n* = 50)	*t*	*P*
Sex [*n* (%)]	Male	22 (44.00)	21 (42.00)	0.023	0.887
	Female	28 (56.00)	29 (58.00)		
Average age (years)		56.26 ± 11.09	55.98 ± 11.13	0.372	0.708
Average duration (days)		3.83 ± 1.15	3.66 ± 1.13	0.459	0.639
Average stone diameter (cm)		1.43 ± 0.46	1.41 ± 0.42	0.454	0.501
Number of common bile duct stone [*n* (%)]	Single	33 (66.00)	34 (68.00)	0.473	0.492
	Multiple	17 (34.00)	16 (32.00)		

**Table 2:** Comparison of operation related indexes (±*s*).

Indicators	Control group (*n* = 50)	Observation group (*n* = 50)	*t*	*P*
Operation time (min)	106.42 ± 15.40	133.58 ± 24.76	6.882	0.000
Incision size (cm)	10.57 ± 1.47	2.45 ± 0.36	10.016	0.000
Blood loss (mL)	206.35 ± 34.22	142.58 ± 21.11	32.623	0.000

**Table 3:** A comparison of the therapeutic benefits of the two groups [*n* (%)].

Indicators	Control group (*n* = 50)	Observation group (*n* = 50)	*χ* ^2^	*P*
Stone clearance rate	49 (98.00)	48 (96.00)	0.503	0.485
Recurrence rate of stones	10 (20.00)	1 (2.00)	4.509	0.033

**Table 4:** Comparison of pain degree (±*s*, score).

Time	Control group (*n* = 50)	Observation group (*n* = 50)
Before the operation	4.72 ± 0.33	4.63 ± 0.46
Three days 3 surgery	3.03 ± 0.26^*∗*^	2.42 ± 0.32^*∗*#^
Three days 7 surgery	2.11 ± 0.36^*∗*^	1.22 ± 0.26^*∗*#^

**Table 5:** Comparison of postoperative recovery (±*s*).

Indicators exhaust time (h)	Control group (*n* = 50)	Observation group (*n* = 50)	*t*	*P*
Eating time (h)	24.33 ± 3.75	20.01 ± 3.70	7.120	0.000
Exhaust time (h)	21.28 ± 4.35	17.80 ± 3.87	6.730	0.000
Out of bed time (h)	46.56 ± 4.71	35.42 ± 5.24	9.903	0.000
Out of bed time (h)	8.55 ± 1.77	5.96 ± 1.28	7.272	0.000

**Table 6:** Comparison of complications [*n* (%)].

Complications	Control group (*n* = 50)	Observation group (*n* = 50)	*χ* ^2^	*P*
Pancreatitis	2 (4.00)	1 (2.00)	—	—
Hyperamylasemia	5 (10.00)	6 (12.00)	—	—
Abdominal cavity infection	4 (8.00)	1 (2.00)	—	—
Bleeding	5 (10.00)	1 (2.00)	—	—
Biliary fistula	1 (2.00)	1 (2.00)	—	—
Total	17 (34.00)	10 (20.00)	6.542	0.014

## Data Availability

The data used to support the findings of this study are available from the corresponding author upon request.
